# Treatment of the Gastroesophageal Reflux Disease with Chinese Herbal Medicine (BanxiaXiexin Decoction): Evidence from Meta-Analysis

**DOI:** 10.1155/2022/1500660

**Published:** 2022-06-15

**Authors:** Jiali Liu, Jinke Huang, Beihua Zhang, Xiaolan Yin, Mi Lv, Zhihong Liu, Fengyun Wang, Xudong Tang

**Affiliations:** ^1^Department of Gastroenterology, Xiyuan Hospital, China Academy of Chinese Medical Sciences, Beijing, China; ^2^Institute of Gastroenterology, Xiyuan Hospital, China Academy of Chinese Medical Sciences, Beijing, China; ^3^Department of Gastroenterology, Peking University Traditional Chinese Medicine Clinical Medical School (Xiyuan), Beijing, China

## Abstract

**Objectives:**

Systematic reviews/meta-analyses (SRs/MAs) are still controversial on the effectiveness of Banxia Xiexin decoction (BXD) to treat gastroesophageal reflux disease (GERD). To assess the evidence reliability and inform the clinical use of BXD, we performed a meta-analysis from previous SRs/MAs to collate, critically appraise, and synthesize the effectiveness of BXD treatment in GERD.

**Methods:**

SRs/MAs were collected by searching major medical databases. The included studies were evaluated in terms of methodological quality and quality of evidence using criteria from the Assessment of Multiple Systematic Reviews 2 (AMSTAR-2) tool, and the Grades of Recommendation, Assessment, Development, and Evaluation (GRADE) system, respectively.

**Results:**

Six SRs/MAs were included in this study. The methodological quality of SRs/MAs was generally unsatisfactory. Unregistered protocols, failure to provide a list of excluded trials, and lack of a comprehensive search strategy were the main limitations of previous SRs/MAs. No high-quality evidence was found to support the effect of BXD on GERD patients. The qualitative data synthesis relied on low-quality trials with a small sample size, which was the main factor for evidence degradation.

**Conclusions:**

BXD seems to have promising efficacy to treat GERD patients. Although the quality of SRs/MAs was generally low and defects were frequent, our study highlights areas where methodologies need to be improved.

## 1. Introduction

The gastroesophageal reflux disease (GERD) is a functional gastrointestinal disorder characterized by heartburn, chest pain, dysphagia, and abdominal pain due to gastric acid entering the esophagus [1]. The global prevalence of GERD has increased substantially—from 424 million in 1990 to 709 million cases in 2017, a change of 67.2% [2]. The GERD imposes a considerable economic burden, driven by the cost of consulting, examining, and prescribing over the countermedications, surgery, and associated complications such as Barrett's esophagus and esophageal adenocarcinoma [3]. The goal of GERD treatment is to relieve or reduce gastric acid secretion, and therefore, antacids, histamine receptor antagonists, and proton pump inhibitors are the main therapeutic drugs [4]. However, the efficacy of conventional drugs varies widely and most of them require long-term or lifelong administration [5]. Moreover, some patients require surgical treatment when conventional treatment is ineffective [4]. As a result, patients often seek complementary and alternative therapies to alleviate their symptoms [6].

The pathogenesis of GERD has not been fully elucidated. According to available evidence, the development of GERD involves a variety of potential mechanisms, such as transient lower esophageal sphincter relaxation, lower esophageal sphincter pressure, hiatus hernia, crural diaphragmatic dysfunction, and impaired esophageal clearance [7]. Pharmacological experiments have verified the effectiveness of Banxia Xiexin decoction (BXD) in the treatment of GERD [8]. Animal experiments have shown that BXD helps to reduce esophageal mucosal injury and decreases the expression of intercellular adhesion molecule-1 and L-selectin [9]. Chronic administration of BXD can increase esophageal sphincter pressure, inhibit gastric acid, and promote the repair of damaged mucosa [10]. In addition, BXD may exert a protective effect on the esophageal mucosa by downregulating the mRNA expression of calponin and caldesmon and regulating the synthesis of calcitonin gene-related peptides to reduce gastric acidity [8]. These available evidence support that BXD has good clinical application prospects, given that it is effective to treat GERD acting in multiple pathways.

Systematic reviews (SRs)/meta-analyses (MAs) are considered the highest level of evidence in evidence-based medicine, yet inconsistent results may interfere with evidence-based decision-making [11,12]. BXD has been widely used in the treatment of GERD in China and is highly effective due to its multicomponent and multitarget characteristics [13]. Numerous SRs/MAs have evaluated the effect of BXD on GERD, but the conclusions of these studies were not consistent, which created a need to ascertain the reliability of previous evidence. Thus, we conducted this overview to systematically evaluate the available evidence for the use of BXD in the treatment of GERD.

## 2. Methods

The protocol of this study was registered in PROSPERO (http://www. crd. York.ac.uk/prospero), and the registration number was CRD42022287497. The methodology was performed following the criteria of the Cochrane Handbook [14].

### 2.1. Search Strategy

Sources of the Cochrane Library, PubMed, Web of Science, Embase, the Chinese database of Chinese Biomedical Database, ChineseVIP, Wanfang, and China National Knowledge Infrastructure were identified from their inception to January, 2022. Gastroesophageal reflux disease, Chinese medicine, Banxia Xiexin decoction, and systematic review were used as search keywords. The strategy used for the PubMed search is shown in Table 1.

### 2.2. Criteria for Considering Studies

Inclusion criteria were as follows: (a) SRs/MAs studies; (b) patients diagnosed with GERD; (c) experimental group treated with BXD and control group treated with Western medicine (WM); and (d) outcomes included effective rate, recovery rate, efficacy under gastroscope, recurrence rate, acid regurgitation, heartburn, and adverse events.

The comprehensive efficacy assessment criteria were as follows [15]: (a) cure: clinical symptoms completely disappeared, gastroscopy showed that the esophageal mucosa was completely restored to normal; (b) effective: clinical symptoms were reduced and gastroscopy showed improvement of esophageal mucosal lesions; and (c) ineffective: clinical symptoms and endoscopy showed no improvement in esophageal mucosal lesions. Effective rate was defined as follows: effective rate = (total number of patients - number of patients with no response)/total number of patients. Efficacy under the gastroscope was classified as follows [16]: (a) cured: gastroscope grade 0 seen by endoscopy; (b) significantly effective: gastroscope grading reduced by more than 2 grades compared with the grade before treatment; but not reaching grade 0; (c) effective: gastroscope grading reduced by more than 1 grade compared with the grade before treatment; and (d) ineffective: gastroscope grading reduced by less than 1 grade, unchanged, or aggravated. Efficacy under the gastroscope was defined as follows: effective rate = (total number of patients - number of patients with no response)/total number of patients. Recurrence was defined as the appearance of clinical symptoms and changes in the gastroscopic esophageal mucosal pathology during the follow-up period in completely cured patients [15]. Recurrence rate was defined as follows: recurrence rate = number of patients with recurrence/total number of follow-up patients.

### 2.3. Exclusion Criteria

Exclusion criteria were as follows: (a) repeated publications; (b) graduate dissertation; and (c) meeting abstracts.

### 2.4. Study Identification

Study identification and data extraction were carried out independently by two authors. Studies were first identified by screening titles and abstracts, after which the full text was read for papers that possibly met the criteria. Items of the included studies were extracted as follows: authors, sample size, interventions, outcomes, relative effect, and main findings.

### 2.5. Quality Assessment

Methodological and evidence quality of the enrolled studies were carried out independently by two authors using the AMSTAR-2 tool and GRADE system, respectively. The methodological quality was ranked as high, moderate, low, or critically low [17]. Evidence quality with GRADE was considered from five aspects (risk of bias, inconsistency, indirectness, imprecision, and publication bias) and given a rating of high to critically low [18].

### 2.6. Data Synthesis and Presentation

A narrative synthesis was performed in this overview. The characteristics and results of each SR/MA as well as the results of AMSTAR 2 were summarized by tabulation. The GRADE evidence profile and summary of findings table were generated by using the GRADE pro GDT online software.

## 3. Results

### 3.1. Literature Screening

The literature search identified 202 relevant records, of which 191 records were removed after screening titles and abstracts. The remaining 11 papers were evaluated through full-text reading. Finally, five records were excluded, and the remaining six SRs/MAs [19–24] met the inclusion criteria (Figure 1).

### 3.2. General Characteristics

Features of included SRs/MAs are outlined in Table 2. All SRs/MAs were written by Chinese researchers and published from 2015 to 2020. The number of enrolled trials ranged from 11 to 31, while the sample size ranged from 914 to 2300. The experimental group received BXD while the control groups received WM.

### 3.3. Methodological Quality Assessment

All included SRs/MAs failed to register protocols and to provide a list of excluded trials. Therefore, previous SRs/MAs were graded critically low for their methodological quality. Furthermore, search strategies, funding source, and conflicts of interest statement displayed different degrees of errors (Table 3).

### 3.4. Evidence Quality Assessment

Due to limitations of the enrolled trails, the evidence strength was weakened for all outcomes. Inconsistency, imprecision, and publication bias also limited the strength of evidence for some outcomes. Four outcomes were deemed of moderate evidence quality, ten outcomes were considered of low quality, and five were of critically low quality. Details are outlined in Table 4.

### 3.5. Results of Meta-Analyses

#### 3.5.1. Effects of BXD on GERD Patients

Two SRs/MAs [19, 23] compared the effects of BXD with those of WM using recovery rate, and the meta-analysis results revealed that the BXD group was superior to the WM group. All SRs/MAs [19–24] compared BXD vs WM using the effective rate as outcome, and the pooled results revealed that the BXD group was also superior to the WM group. Efficacy under the gastroscope was reported in four studies [19–21, 24]; three of which [19, 21, 24] showed that the BXD group was superior to WM-treated patients. The other study [20] reported no significant differences between these two groups. Four SRs/MAs [19, 21, 22, 24] compared BXD and WM using the recurrence rate of GERD; three of which [19, 22, 24] showed that the BXD group was superior to the WM group, while one study [21] found no significant difference between these two groups. In addition, BXD was reported to be superior to WM in relieving heartburn, but showed no advantage in relieving acid reflux [21].

#### 3.5.2. Safety of BXD for GERD

The pooled results of adverse events were reported in only one study [20], and the results showed that there was no statistical difference between BXD and WM groups.

## 4. Discussion

SRs/MAs are considered the highest level of evidence in evidence-based medicine [11]. However, low quality SRs/MAs may instead mislead decision makers [25]. Therefore, to collate, critically appraise, and synthesize the clinical evidence of the use of BXD to treat GERD, we conducted an overview of previous SRs/MAs on the matter.

After a systematic review and synthesis, it was found that the gap between evidence and its implementation in clinical practice stems from the low quality and uncertain characteristics of previous evidence. There are several notable findings from this study. First, all included SRs/MAs were published in recent years (2015 to 2020), suggesting that BXD is starting to gain attention as a complementary alternative therapy for GERD. Second, based on results from the AMSTAR-2 tool and the GRADE system, the methodological and evidence qualities of the included studies were limited, which means current evidence cannot provide a reliable basis for clinical decision-making. Third, almost all SRs/MAs yielded positive results. Of note, most authors did not tend to draw firm conclusions about the effects of BXD on GERD patients due to small sample size and low quality of randomized controlled trials.

The AMSTAR-2 tool highlighted several challenges of SRs/MAs that should be addressed. First, studies did not register their protocols. The pre-registration protocol helps to improve transparency, minimize potential risk of bias, reduce duplicated work, and keep the study up to date. It is advocated and recommended that authors register protocols in public databases such as PROSPERO to avoid the risk of bias. Second, authors did not account for publication bias when selecting literature for their SRs/MAs. Therefore, SRs/MAs should provide a comprehensive search strategy for all databases, as a comprehensive and precise search helps to avoid the inclusion of ineligible studies and reduces the risk of publication bias. Furthermore, a list of excluded trials and exclusion criteria improves transparency and can be presented by direct reference or as a supplementary file. Finally, funding sources should be fully reported, as results from commercially funded research might be biased toward funders. Based on the GRADE system, the risk of bias of the enrolled trials was the most common downgrading factor, indicating that the main cause of the reduced quality of evidence came from the quality of the original trials. Only well-designed and rigorously conducted trials can reduce or avoid bias. Specific methods of randomization should be clearly described to reflect whether randomization has been successfully achieved. Moreover, the allocation concealment and blinding method should be fully reported, while large sample sizes and high-quality trials are the basis for high-quality evidence sources.

Numerous SRs/MAs have evaluated the use of BXD to treat GERD, but the quality of these studies is limited and their results are not fully consistent, which is not conducive to the use their evidence. Compared with traditional SRs/MAs, an overview facilitates a comprehensive evaluation of current evidence on multiple identical topics, provides more focused high-quality evidence, and identifies key flaws in evidence use. To our knowledge, this is the first overview of SRs/MAs exploring the effect of BXD on GERD patients using AMSTAR-2 and GRADE. Results herein presented on the methodological and evidence qualities of previous SRs/MAs might help to inform evidence-based decision making and guide future high-quality studies [27, 28].

Some limitations must be acknowledged. First, SRs/MAs lacked detailed characteristics of participants and observation time points. These can hinder the analysis and interpretation of data and reduce the translation of evidence into clinical practice. Second, only eight commonly used public databases were searched in this study. There might be eligible literature in other databases, which were not identified, thus limiting the comprehensiveness of this study. Furthermore, the on standards used in each included study were not fully reported, so it was not possible to determine if they were suitable to be reported together on effectiveness. Future studies are recommended to fully report the details of the inclusion criteria to minimize any potential risk of bias.

## 5. Conclusion

BXD seems to have a promising efficacy in the treatment of GERD patients. Although the quality of included SRs/MAs was generally low and defects were frequent, our study highlights areas where methodologies need to be improved.

## Figures and Tables

**Figure 1:** Literature screening flowchart.

**Table 1:** The search strategy for PubMed.

Query	Search term
#1	Gastroesophageal reflux (mesh)
#2	Gastroesophageal reflux (Title/Abstract) or gastroesophageal reflux disease (Title/Abstract) or Gastric acid reflux (Title/Abstract) OR gastro-oesophageal reflux (Title/Abstract) or gastroesophageal reflux (Title/Abstract) or Barrett esophagus (Title/Abstract) or esophagitis (Title/Abstract)
#3	#1 OR #2
#4	Traditional Chinese medicine (mesh)
#5	Chinese medicine (Title/Abstract) or Banxia Xiexin decoction (Title/Abstract) OR herbal medicine (Title/Abstract)
#6	#4 OR #5
#7	Meta-analysis as topic (mesh)
#8	Systematic review (Title/Abstract) or meta-analysis (Title/Abstract) or meta-analysis (Title/Abstract) or meta-analyses (Title/Abstract) or meta-analysis (Title/Abstract)
#9	#7 OR #8
#10	#3 AND #6 AND #9

**Table 2:** General characteristics of the included reviews.

Studies	Diagnosticcriteria	Trials (subjects)	GERD Classification	Experimental Intervention	Control Intervention	Duration	Follow-up period	Quality assessment	Results summary
Yu [19]	①, ②	13 (1089)	NERD, RE	BXD	WM	4–8 weeks	NA	Cochrane Criteria	BXD was more effective to treat GERD than the optimal combination of WM.
Chen [20]	NA	24 (2002)	NERD, RE	BXD	WM	Unclear	NA	Jada scale	BXD was superior to WM alone in the treatment of GERD, but there was no significant difference in gastroscopy results or on the occurrence of adverse reactions.
Dai [21]		31 (1210)	NERD, RE	BXD	WM	4 weeks- 8 months	NA	Cochrane Criteria	BXD showed a potential benefit to GERD patients, but further research is needed due to methodological quality and sample size limitations.
Zheng [22]	NA	11 (1305)	NERD, RE	BXD	WM	4–8 weeks	NA	Cochrane Criteria	BXD treatment improved total effective and recurrence rates for GERD as compared with those of the control group．
Qi [23]	NA	27 (2300)	NERD, RE	BXD	WM	4–8 weeks	3 or 6 months	Cochrane Criteria	The use of BXD tin the treatment of GERD was superior to WM alone in terms of cure rate and total effective rate.
Guo [24]	NA	12 (914)	NERD, RE	BXD	WM	4–8 weeks	NA	Cochrane Criteria	BXD was superior than conventional WM to treat GERD without inducing severe adverse reactions.

①: Consensus Opinion on GERD in China [25]; ②: Chinese Herbal Medicine New Medicine ClinicalResearch Guiding Principle [26]. BXD : Banxia Xiexin decoction; NERD: nonerosive reflux disease; RE: reflux esophagitis; WM : Western medicine; NA: not applicable.

**Table 3:** Results of the AMSTAR-2 assessments.

Author, Year	AMSTAR-2																Quality
	Q1	Q2	Q3	Q4	Q5	Q6	Q7	Q8	Q9	Q10	Q11	Q12	Q13	Q14	Q15	Q16	
Yu [19]	Y	PY	Y	PY	Y	Y	N	Y	Y	Y	Y	Y	Y	Y	Y	Y	CL
Chen [20]	Y	PY	Y	Y	Y	Y	N	Y	Y	Y	Y	Y	Y	Y	Y	Y	CL
Dai [21]	Y	PY	Y	Y	Y	Y	N	Y	Y	Y	Y	Y	Y	Y	Y	Y	CL
Zheng [22]	Y	PY	Y	PY	Y	Y	N	Y	Y	N	Y	Y	Y	Y	Y	N	CL
Qi [23]	Y	PY	Y	PY	Y	Y	N	Y	Y	N	Y	Y	Y	Y	Y	N	CL
Guo [24]	Y	PY	Y	PY	Y	Y	Y	Y	Y	Y	Y	Y	Y	Y	Y	Y	CL

Y : Yes; PY: partial Yes; N : No; CL : Critically low; L : Low; H : High.

**Table 4:** Results of evidence quality.

Studies	Outcomes	Limitations	Inconsistency	Indirectness	Imprecision	Publicationbias	Relative effect(95% CI)	Quality
Yu [19]	Recovery rate	−1	0	0	0	0	RR 1.55 (1.17, 2.05)	M
	Effective rate	−1	0	0	0	0	RR 1.15 (1.10,1.21)	M
	Efficacy under gastroscope	−1	0	0	0	0	RR 1.21 (1.09, 1.35)	M

Chen [20]	Recurrence rate	−1	0	0	−1	0	RR 0.25 (0.09, 0.72)	L
	Effective rate	−1	0	0	0	0	OR 3.96 (2.96, 5.28)	M
	Efficacy under gastroscope	−1	0	0	−1	0	OR 1.99 (0.99, 3.65)	L
	Adverse events	−1	−1	0	0	−1	OR 0.26 (0.06, 1.07)	CL

Dai [21]	Effective rate	−1	0	0	0	−1	OR 3.25 (2.15, 4.94)	L
	Efficacy under gastroscope	−1	−1	0	0	0	OR 1.96 (1.21, 3.18)	L
	Acid regurgitation	−1	−1	0	0	0	SMD 0.51 (-0.90, 1.92)	L
	Heartburn	−1	−1	0	0	0	SMD -0.68 (-1.25, -0.12)	L
	Recurrence rate	−1	−1	0	−1	0	OR 0.35 (0.11, 1.16)	CL

Zheng [22], 2016	Effective rate	−1	−1	0	0	0	OR 4.16 (2.91,5.59)	L
	Recurrence rate	−1	−1	0	0	0	OR O.27 (0.15,0.48)	L

Qi[23], 2016	Effective rate	−1	−1	0	0	−1	OR 3.31 (2.57,4.27)	CL
	Recovery rate	−1	−1	0	−1	−1	OR 1.88 (1.53, 2.31)	CL

Guo[24], 2015	Effective rate	−1	0	0	0	−1	OR 3.41 (2.22, 5.23)	L
	Efficacy under gastroscope	−1	0	0	−1	−1	OR 1.58 (1.04, 2.41)	CL
	Recurrence rate	−1	0	0	0	−1	OR 0.23 (0.14,0.40)	L

-1: downgrade; 0: not downgrade; CL: critically low; L : Low; M: moderate; RR: relative risk; OR: odds ratio; SMD : SMD: standardized mean difference.

## Data Availability

All analyses were based on previously published studies.

## Abbreviations

BXD: Banxia Xiexin decoction
GERD: Gastroesophageal reflux disease
SR: Systematic review
MA: Meta-analysis
AMSTAR-2: Assessment of multiple systematic reviews 2
GRADE: Grading of recommendations, assessment, development, and evaluation
WM: Western medicine.
